# Discontinuous Track Recognition System Based on PolyLaneNet for Darwin-op2 Robot

**DOI:** 10.1155/2022/5431886

**Published:** 2022-02-01

**Authors:** Xi-Bao Wu, Si-Chuan Lv, Xiao-Hao Wang, Shi-Zhuo Zhang, Qiong Liu, Yi-Qun Wang, Wen-bai Chen

**Affiliations:** School of Automation, Beijing Information Science and Technology University, Beijing, China

## Abstract

This paper proposes and demonstrates a single-line discontinuous track recognition system by associating the track recognition problem of a humanoid robot with the lane detection problem. The proposal enables the robot to achieve stable running on the single-line discontinuous track. The system consists of two parts: the robot end and the graphics computing end. The robot end is responsible for collecting track information and the graphics computing end is responsible for high-performance computing. These two parts use the TCP for communication. The graphics computing side uses PolyLaneNet lane detection algorithm to train the track image captured from the first perspective of the darwin-op2 robot as the data set. In the inference, the robot end sends the collected tracking images to the graphics calculation end and uses the graphics processor to accelerate the calculation. After obtaining the motion vector, it is transmitted back to the robot end. The robot end parses the motion vector to obtain the motion information of the robot so that the robot can achieve stable running on the single-line discontinuous track. The proposed system realizes the direct recognition of the first perspective image of the robot and avoids the problems of poor stability, inability of identifying curves and discontinuous lines, and other problems in the traditional line detection method. At the same time, this system adopts the method of cooperative work between the PC side and the robot by deploying the algorithm with high computational requirements on the PC side. The data transmission is carried out by stable TCP communication, which makes it possible for the robot equipped with weak computational controllers to use deep-learning-related algorithms. It also provides ideas and solutions for deploying deep-learning-related algorithms on similar low computational robots.

## 1. Introduction

The humanoid robot track and field project mainly requires the robot to reach the end point in the shortest time through various trajectories without human control. The evaluation criteria mainly include the passing time of the robot, the correct movement along the trajectory direction, and the recognition effect of obstacles on the trajectory. Common track and field runways are single continuous line and curve, double continuous line and curve, single discontinuous line and curve, double discontinuous line and curve, etc. Some tracks also include up and down slopes, up and down stairs, obstacles, crossroads, and other elements, which greatly tests the comprehensive technical level of robots and their teams. Our design focuses on identifying single continuous and discontinuous trajectories captured by first-person robots. In essence, the track recognition of humanoid robot in track and field competition is mainly to identify one or several lines in the picture captured by the first person of the robot. These lines have different colours, continuous state, intersection, and other characteristics, which play a guiding role in the movement of robots, similar to the track line of human track and field competition and the lane line of vehicles driving on the road. The robot uses various algorithms to identify the track and obtains the offset position and guiding direction of different forms of track. Then, the postprocessing analysis is carried out on the offset position and orientation direction of the trajectory to determine the motion direction of the robot at the next moment, using a fixed step to modify the lateral offset of the movement or directly providing a direction vector.

There are many kinds of track recognition algorithms for humanoid robot track and field competitions. The simplest algorithm is the recognition method based on photoelectric sensor, which uses the colour difference between the track line colour and the track bottom colour to identify. Some of the complex algorithms are various visual algorithms based on cameras. The camera deployed on the robot captures the first person or non-first-person real-time images of the robot for recognition, including traditional recognition algorithms such as pixel-by-pixel comparison method, Hough [1] transform method, connected domain recognition method, line segments angles computation [2], and deep learning recognition algorithms [3–14] such as deep convolutional neural network recognition algorithm. In the track and field competition of humanoid robot, single-line or double-line noncontinuous track is often more difficult to identify than continuous track. In order to solve the problem of rapid and accurate recognition of single-line noncontinuous track by robots, this paper comprehensively examines various visual recognition algorithms and nonvisual recognition algorithms, combined with the lane line detection algorithm PolyLaneNet [15]; a deep learning algorithm is deployed on the humanoid robot with low computing power, so that it can accurately identify the track line in the track and field competition of humanoid robot, so as to achieve the effect of high-level competition.

PolyLaneNet algorithm constructs the recognition problem of lines into the task of polynomial formula analysis of lines. Common lanes or racetracks can be resolved as an N-order polynomial (N is the natural number). PolyLaneNet first puts the image into the deep convolutional neural network (one of EfficientNet [16, 17], ResNet34 [18], ResNet50, and ResNet101) for feature extraction and then the extracted features are postprocessed to obtain the polynomial formula that can accurately describe the line. It ensures high recognition accuracy and has high computing speed. The PolyLaneNet algorithm was originally used to solve the lane line detection problem. Because the lane line recognition problem in humanoid robot track and field competition is similar to the lane line detection problem and even in most cases it is simpler than the lane line problem (reducing the occlusion of the lane line by the side car, there are many lanes, there are many types of lane lines, and the lane line is thicker and more obvious than the lane line and it is easier to identify), this paper will transplant the PolyLaneNet algorithm with excellent performance in the lane line detection problem to the track recognition problem of humanoid robot track and field competition.

The single-line noncontinuous track recognition system designed in this paper consists of two parts: the robot end and the graphics computing end. The graphics computing end is composed of a computer or GPU (graphics processing unit) server containing an independent graphics computing card. After the robot camera captures the real-time picture, the picture is transmitted to the graphics computing end through TCP (Transmission Control Protocol) communication. The graphics computing end performs PolyLaneNet algorithm reasoning on the real-time picture received by TCP communication and processes the reasoning results to obtain the direction vector that the robot should move next. The direction vector is transmitted back to the robot through TCP communication. The robot receives the direction vector and controls the steering gear to move. The average speed and recognition stability of darwin-op2 robot in this scene have been significantly improved. Specifically, the darwin-op2 robot runs stably on the track and field track at its own 0.5 times speed (actual 0.12 m/s) and 0.7 times speed (actual 0.15 m/s), which meets the running requirements of the robot on the track and field track. And the robot performed well even at full speed, only occasionally running out of the field. Good performance has been achieved in many experiments and controls.

## 2. Relevant Algorithms

### 2.1. Track Line Recognition Algorithms

In the humanoid robot track and field race, the teams used various methods to identify the track line. The following will introduce several common recognition methods in humanoid robot track and field competition.

To begin with, the first recognition method is based on a photoelectric sensor. The photoelectric sensor has a light intensity receiving terminal, which can convert the received light intensity into an electrical signal with analog value. Due to the difference between the colour of the track line and the background colour of the track in the race, the reflected light intensity is different and the analog value converted into electrical signal is also different. The recognition algorithm based on photoelectric sensor uses the above principle to recognize the track line and distinguishes the track line from the track background by distinguishing different simulation value intervals. The disadvantage of this recognition method is that it is easily affected by the external light intensity environment, the threshold changes greatly, and the generalization ability of different light conditions is weak. It needs to adjust the sensor threshold before each race. And because of the characteristics of the sensor itself, it cannot support the rapid movement of the robot and cannot recognize the discontinuous track.

The second pixel-by-pixel comparison method is based on camera. Firstly, the image captured by the camera is preprocessed by Gaussian filtering, binarization, expansion, and corrosion to get a binarization image, where the track line is white and the background is black or the track line is black and the background is white. Then, the pixels of the binary image are traversed according to a certain rule and the pixel position of the track line in the picture is obtained. The disadvantage of this algorithm is that it is easy to form false recognition to the noise or large area colour block after image preprocessing; also, the recognition effect of discontinuous track is poor.

Furthermore, the connected domain recognition algorithm based on camera is used frequently. Firstly, the image captured by the camera is preprocessed by Gaussian filtering, binarization, expansion, and corrosion to get a binary image. Then, the connected domain of the binary image is identified and the largest connected domain is the track line. The lateral offset, inclination angle, and other information of the track line can be obtained by calculating the connected domain. The algorithm still cannot eliminate the interference of large area colour block and the recognition effect of discontinuous track is also poor.

The Hough transform algorithm based on camera is also one of recognition methods. The image is preprocessed by Gaussian filtering, edge detection, and binarization. Then, the image is mapped from the Cartesian coordinate system to the polar coordinate system. The algorithm takes the local maximum value, sets the threshold, and filters the noise for each point in the polar coordinate system. Finally, the points in polar coordinate system are transformed back to Cartesian coordinate system, which is the straight line in the original image recognized by the algorithm. This algorithm can identify the interference of discontinuous track, immune noise, and large-area colour blocks and has strong recognition ability for straight lines. However, it is easy to form false detection for long strip interference and has weak recognition ability for curves.

### 2.2. Lane Detection Algorithms

The common methods of track line identification described above all have defects in different aspects. In this paper, we notice that the recognition of track lines in humanoid robot track and field events is essentially to find or fit one or more long lines in an ROI (region of interest) region of the image, which is used to guide the robot to a certain direction. The problem of lane detection in the field of automatic driving is essentially to find or fit the lane in an ROI region of the image, which is used to guide the car to a certain direction. At the same time, the lane detection is similar to the track recognition; there are continuous line and discontinuous line, different degrees of noise interference and occlusion, and real-time problems. Therefore, this paper considers that the problem of track line recognition in humanoid robot track and field events and the problem of lane line detection in automatic driving are essentially the same kind of problems. They are all used to identify one or more lines in the ROI region to guide the direction of movement, which can be solved by the same or similar methods. The problem of lane detection takes the colour picture as the input and the image segmentation examples, some points, or parameters as the output. This paper summarizes some common lane detection methods as follows.

The traditional lane detection algorithm is mainly based on Hough transform and the detection method is the same as the Hough transform detection method mentioned above. In recent years, with the rapid development of deep learning and the continuous success of convolutional neural network in many computers vision tasks, various research teams gradually move the solution of lane detection problem closer to the deep learning method. At present, several commonly used lane detection methods based on deep learning mainly include detection method, grid method, polynomial regression method, and anchor-based detection method.

Detection methods mainly include Lanenet [19], Scnn [20], Sad, and so on. Lanenet algorithm is a classic algorithm and it is widely used in industry. It belongs to instance segmentation algorithm, but its disadvantage is that it relies on clustering and the detection result is unstable. Scnn algorithm is a semantic segmentation algorithm, which uses the method similar to RNN to learn the spatiotemporal information. It defines K lines in advance, makes K classification prediction for each pixel, and finally combines the points with the same results to get the lane lines to be detected, but the disadvantage is that the recognition speed is slow. Sad algorithm is also a segmentation algorithm; its structure is lighter than Scnn algorithm, so the recognition speed is faster than the Scnn algorithm, but the recognition accuracy is relatively low.

The main idea of the gridding method is to turn the pixel problem of the image into a cell problem, which is similar to the idea of downsampling. The recognition speed is faster, but because it is equivalent to reducing the resolution of the image, the recognition accuracy of the algorithm is low.

Polynomial regression method is to fit the lane line into an n-order polynomial (n is a natural number). The speed of recognition is faster, but the disadvantage of the polynomial regression method is that it relies on a priori and has low flexibility in complex scenes

The detection method based on anchor point is similar to the target detection method. Some lines with various angles are defined in advance and their offsets are learned. This detection method also depends on a priori and has low flexibility in complex scenes.

## 3. Algorithm Selection

### 3.1. The Original Algorithm

Before carrying the track line recognition algorithm used in this design, the track line recognition algorithm used by our team is the pixel-by-pixel comparison method based on the camera mentioned above.

First, a camera is used to capture an image of the robot from the first view. Then, the image is transformed from a three-channel colour image to a single-channel grey image and the grey image is binarized according to a certain threshold (the threshold needs to be adjusted manually according to the colour and illumination of the competition venue), so as to change the colour of the track into black and the colour of the track line into white. The transformation process is shown in Figure 1.

Then, the binary image is divided into two regions (the height range of the region is adjustable) and the two regions are compared pixel by pixel to find the track line. After the lateral offsets of the track lines in the upper and lower regions are obtained, the weighted sum of the two lateral offsets and the offset are added based on some decision-making methods. The final offset is the lateral offset that the robot needs to move forward at the next moment.

The specific process of pixel-by-pixel comparison is to traverse the pixels of each region from top to bottom. For each row of pixels, traverse from the middle to both sides. When three consecutive white pixels are encountered, it is the track line that meets white (after binarization). The abscissa position of the pixel is recorded and stored in the array. After the end of line-by-line traversal, the abscissa of the white track line found in each line and stored in the array is averaged and then the abscissa of the middle point in the image is subtracted to get the average lateral offset of the current area track. If there is no track in the current area, the lateral offset is 0. The time complexity of this method is O (*n*^2^).

The pixel-by-pixel comparison method based on camera has simple logic and short time consumption, but it compares the pixels, only identifies the local, and then combines the results of local recognition to form a global decision. The disadvantage of local recognition is that it is easy to be interfered by noise and large area colour block (as shown in Figure 2). Once there is interference in the picture which is far away from the real track line, the final global decision will be inaccurate. Because of its line-by-line recognition of pixels and small track area (generally speaking, the camera only captures a small part of the track in front of the robot), once it encounters a discontinuous track line, it will not find the track line.

### 3.2. The PolyLaneNet Algorithm

In order to reduce or eliminate the noise and large area colour block interference and realize the recognition of discontinuous track, we need an algorithm to recognize the global information and increase the area of the track captured by the robot first person picture. Common algorithms such as Hoff transform map Cartesian coordinate system to polar coordinate system, reorganize all local information, then carry out local recognition in polar coordinate system and use global information in disguised way, eliminate noise and nonlong bar colour block interference, and realize recognition of discontinuous linear track, but they cannot recognize curve track better. Convolution neural network can recognize local information and global information by using many convolutions check images for several times and extract higher dimension features, which can fully satisfy the interference of noise and large area colour block and can recognize not only discontinuous linear track, but also discontinuous curve track, The ability of anti-jamming is enhanced and the ability of track line recognition is improved. The disadvantage is that the calculation is large and a large amount of data is needed to train the model. After considering several methods mentioned above, this paper finally decides to use the method of deep learning (deep convolution neural network) to identify the track line. The method of deploying the model on PC (personal computer) and communicating with robot through wireless LAN (local area network) solves the problem that the computer human controller cannot bear the convolution neural network calculation.

The previous paper lists several different principles and effects of lane detection methods based on deep learning. Compared with lane detection in automatic driving, the scene of track line recognition in humanoid robot track and field race is simpler (as shown in Figure 3), but it requires higher real-time performance. Therefore, this paper selects polynomial regression method, which has faster recognition speed and higher recognition accuracy, but higher requirements for scene environment. The PolyLaneNet (lane estimation via deep polynomial regression) algorithm proposed in 2020 is an excellent polynomial regression algorithm in lane detection. The theoretical FPS (frames per second) of the algorithm is up to 115 and the accuracy of the algorithm is up to 93% in TuSimple data set. If it is transplanted to the track line recognition of humanoid robot track and field race, its high FPS can reduce the time cost and improve the real-time performance as much as possible and the simpler scene in the track line recognition also reduces the false detection and missing detection rate of the algorithm and ensures the accuracy of the recognition. Therefore, this paper uses PolyLaneNet algorithm to identify the track line.

## 4. Algorithm Design Based on PolyLaneNet

### 4.1. Principle Overview

In practical application, there are many problems in the recognition of lane line or track line in track and field competition, such as occlusion, wear, discontinuous line, and so on. The shape of the line is thin and long, which leads to sparse supervision signal, which is difficult to detect. At the same time, the task requires high real-time. Based on convolutional neural network, the PolyLaneNet algorithm used in this paper uses ResNet series network or EfficientNet network as backbones to extract features from images. The extracted features pass through a layer of full connection layer to get several one-dimensional vectors; each vector contains the information of the highest point, the lowest point of a line in the graph confidence information and polynomial coefficient information. The algorithm structure is shown in Figure 4.

PolyLaneNet expects as input images taken from a forward-looking vertical camera, and outputs, for each image, *M*_max_ lane marking candidates (represented as polynomials), as well as the vertical position *h* of the horizon line, which helps to define the upper limit of the lane markings. The architecture of PolyLaneNet consists of a backbone network (for feature extraction) appended with a fully connected layer with *M*_max_ + 1 outputs, being the output 1,…, *M*_max_ for lane marking prediction and the output *M*_max_ + 1 for *h*. PolyLaneNet adopts a polynomial representation for the lane markings instead of a set of points. Therefore, for each output *j*, *j* = 1,…, *M*_max_, the model estimates the coefficients *p*_*j*_ = *{a*_*k,j*_*}*^*K*^_*k*_ = 0 representing the polynomial, shown as follows:

(1) $$\begin{array}{c} p_{j}\left(y\right)=\sum_{k=0}^{K}a_{k,j}y^{k}, \end{array}$$

where *K* is a parameter that defines the order of the polynomial. As illustrated in Figure 4, the polynomials have restricted domain: the height of the image. Besides the coefficients, the PolyLaneNet estimates, for each lane marking j, the vertical offset sj, and the prediction confidence score *c*_*j*_∈[0, 1]. In summary, the PolyLaneNet model can be expressed as follows:

(2) $$\begin{array}{c} f\left(I;\theta \right)=\left({\left\{p_{j},s_{j},c_{j}\right\}}_{j=1}^{M_{max}},h\right), \end{array}$$

where *I* is the input image and *θ* is the model parameters. At inference time, as illustrated in Figure 4, only the lane marking candidates whose confidence score is greater than or equal TO a threshold are considered as detected.

### 4.2. Backbone Process

The original meaning of backbone is human backbone and then extended to the meaning of pillar, core, and so on. Backbone represents the foundation of the whole model in deep learning, because the subsequent tasks such as classification, detection, and generation are based on the extracted features, so in the visual field, backbone is the process of image feature extraction. In the field of machine vision, depth convolution neural network is mainly used to extract image features. Convolution neural network uses convolution check image of specified size to convolute and obtains image texture and other features and then uses these features for various postprocessing. Convolution neural network uses back propagation, gradient descent, and other methods to learn and update the parameters of convolution kernel and the weight parameters of convolution kernel do not need to be adjusted manually. Due to the strong nonlinear modelling ability of neural network, convolutional neural network can solve most problems in many application scenarios. The basic structure of convolutional neural network is shown in Figure 5.

PolyLaneNet algorithm takes ResNet series network or EfficientNet series network as the backbone of the model for feature extraction. ResNet network and EfficientNet network belong to deep convolution neural network. The ResNet series network realizes the deeper development of the network through the “residual unit,” which enables the network to recognize more advanced features. The EfficientNet series network comprehensively improves the depth, width, and resolution of the input image of the network and uses the network structure search method to search the network structure, so as to obtain the results of low resource consumption, high efficiency, and low-cost network with high recognition accuracy.

### 4.3. Posttreatment Process

The input image is transformed into a one-dimensional vector with the length of (6 *∗* *n* + 1) after feature extraction by the depth convolution neural network in the backbone. We transform it into a two-dimensional feature of 7 *∗* *n* (7 one-dimensional vectors) for output, which contains the information of *N* lines. The information of each line includes four polynomial coefficients, one ordinate of the lowest point, one ordinate of the highest point, and one confidence level. After several steps of postprocessing, we need to use an array of points to represent the recognized line.

First of all, we filter out the vector that does not recognize the line (the vector with the confidence of 0) and leave the vector that recognizes the line (because this system does single track identification, only the vector with the highest reliability is retained). Then, we traverse these vectors, extract the vertical axis coordinates of the highest point and the lowest point of each line, construct an array of 100 based on the two vertical coordinates, and divide its height into 100 equal parts. Then, we fit the line according to the four polynomial coefficients and the array with a length of 100 and combine the abscissa calculated with the ordinate divided into 100 parts to form 100 coordinates, which represent the specific shape of the line we fit.

Finally, the decision-making process of the fitted line is carried out. We take the highest point, the middle point, and the lowest point to calculate the weighted difference and get the direction vector which needs to control the robot at the next moment and send it to the robot through TCP communication.

The whole postprocessing flow chart is shown in Figure 6.

## 5. Realization of the Discontinuous Track System

### 5.1. System Flow

Because the computing power of cm740, the core control board of darwin-op2 robot, is not enough to support PolyLaneNet algorithm for reasoning, the gtx1650 super graphics card on PC is used for model reasoning. The information transmission between robot and PC is supported by wireless LAN.

The single-line discontinuous track recognition system of the whole robot consists of discontinuous track, robot, PC terminal, and a local area network, as shown in Figure 7.

Because the communication between robot and PC requires high stability and UDP (User Datagram Protocol) communication has the problem of packet loss, we choose more stable TCP communication instead of UDP communication.

The whole operation process of the system is as follows:

- The robot and PC handshake in LAN to establish TCP communication.
- The robot camera captures the single track picture from the first perspective, packages the picture into a socket package, and transmits it to the PC through TCP communication.
- After receiving the socket packet, the PC transcodes the data into pictures.
- On the PC side, the transcoded image is put into the PolyLaneNet algorithm for forward reasoning and N one-dimensional vectors are obtained after feature extraction by backbone.
- The PC end carries on the postprocessing to the N one-dimensional vectors obtained from the forward reasoning, fits the array which can represent the track line, and extracts the coordinates of the highest point, the middle point, and the lowest point of the track line.
- The PC end calculates the coordinates of the highest point, middle point, and lowest point of the extracted track line, obtains the direction vector of the track line (that is, the direction vector that the robot needs to move at the next moment), and packages it into a socket package, which is sent to the robot through TCP communication.
- After receiving the socket packet, the robot transcodes the data into an array vector and transmits the value of the vector to the API that controls the robot to run in the specified direction.
- At the next moment, the robot camera will continue to capture the single track picture from the first perspective and repeat steps 2–7.

The operation flow chart of the system is shown in Figure 8.

### 5.2. Data Set

In this paper, 3141 images with common floor as the track and 5 cm purple line as the track line are collected and the RGB three channels are rearranged and combined and a data set of 18846 images is obtained. The data set is shown in Figure 9.

On the PC side, the image is first scaled to 640 *∗* 360 for saving and the data set is shown in Figure 9. Then, the image is annotated with “Label Me” annotation software. Each picture is marked with 7 points to represent the track line, as shown in Figure 10.

## 6. Results and Optimization

### 6.1. Preliminary Results

The system is tested on a green track and 5 cm wide white track. In order to ensure the stability of recognition, the half speed of the normal speed (0.24 m/s) of the robot is used to test and the average speed is about 0.11 m/s. The average speed is about 0.14 m/s and the recognition stability is poor. Finally, the normal speed is used to test, the average speed is about 0.15 m/s, and the recognition stability is very poor. The FPS of the system in three cases is always 6–9. The experimental results are summarized in Table 1.

### 6.2. Increasing the FPS of the System

According to the preliminary results, it can be seen that the FPS of the system is very low, which leads to the slow reaction speed of the robot, resulting in its frequent off track. This problem can be alleviated and solved by reducing the movement speed of the robot and the time consumption in the system program. The generalization ability of the system is poor and the robot can only recognize the green track and white track line. If the colour of the track or track line is changed, the robot cannot recognize it. This problem can be solved by using more data sets for training and normalizing the colour of the screen.

Because the ultimate goal of humanoid robot track and field competition is to reach the destination with the fastest speed and reducing the robot's movement speed can enhance the stability, but it is contrary to the ultimate goal, this method can cure the symptoms but not the root cause. Therefore, it is necessary to improve the system FPS by reducing the time consumption of the system program. Through the separate detection of the time consumption of each process of the system, it is found that the most time-consuming process is the TCP communication transmission picture part, the postprocessing part of the PC algorithm, and the control part of the robot movement. Because the part that controls the robot's movement calls the underlying API directly, it cannot be optimized, so this paper attempts to optimize the TCP communication part and the algorithm postprocessing part.

In this paper, the main details of the screen are not lost and the recognition accuracy rate is not affected. Firstly, the image is reduced from 320 *∗* 240 to 40 *∗* 22 resolution and then packaged into socket packet for transmission. This greatly reduces the amount of data when TCP communication transmits the picture, thus greatly shortening the transmission time.After the image is compressed, the proportion can be reduced by half. While the main information of the image is retained, the data quantity changes to 0.01146 times of the original, which makes the time consuming of transmission picture greatly reduced.

The results after system optimization are shown in Table 2.

It can be seen that the average speed, recognition stability, and system FPS of the robot in this scene have been significantly improved, which meets the requirements of the robot running on the track and field track.

## 7. Conclusions

This design uses the method based on deep learning (deep convolution neural network) to detect the single line, curve, continuous, and discontinuous track line in humanoid robot track and field race. It is found that the essence of the track line detection problem in humanoid robot track and field race is the same as that in automatic driving. Therefore, the solution of lane detection in automatic driving is applied to the problem of track detection in humanoid robot track and field events. The high-FPS and high-precision PolyLaneNet model is selected to detect the single track continuous and discontinuous track lines in track and field events. Thanks to the strong nonlinear modelling ability of deep neural network, the system can recognize the first-person image of robot directly and avoid all kinds of problems in traditional line detection methods (poor stability, unable to recognize curves, discontinuous lines, etc.). However, due to the limited computing power of the cm740 controller of darwin-op2 robot, it is unable to directly carry the deep neural network. Therefore, this system uses the method of working with the robot on the PC side, deploys the PolyLaneNet algorithm with high computing power demand on the PC side, uses the LAN to connect the PC side and the robot, and transmits data through stable TCP communication. It makes it possible for darwin-op2 robot equipped with weak computing power controller to use deep learning correlation algorithm and also provides ideas and solutions for deploying deep learning correlation algorithm on similar low computing power robots.

Subsequently, we will solve the problem of noise in the result vector obtained by the PolyLaneNet algorithm of the picture captured by the camera due to strong jitter during robot running and we can alleviate and solve the problem by using Kalman filter and other methods for the result vector obtained by the PolyLaneNet algorithm. Using dynamic information, Kalman filter can not only filter out the noise caused by picture jitter, but also predict the guidance direction of the track line at the next moment. Theoretically, it can alleviate the noise problem caused by strong picture jitter to a certain extent.

## Figures and Tables

**Figure 1:** Image processing by pixel comparison method: original image (a), grey image (b), and binary image (c).

**Figure 2:** Image processing with noise and colour block: original image (a), grey image (b), and binary image (c).

**Figure 3:** Lane detection pending image (a) and track detection pending image (b).

**Figure 4:** PolyLaneNet structure diagram.

**Figure 5:** Basic structure of convolutional neural network.

**Figure 6:** Postprocessing flow.

**Figure 7:** Schematic diagram of track and field competition between the robot and PC.

**Figure 8:** System flow chart.

**Figure 9:** Filtered and scaled data set.

**Figure 10:** Labeling data sets.

**Table 1:** Summary of experimental results.

Theoretical velocity	Actual average speed	Off track times	FPS
0.5 times speed	0.11 m/s	1	6–9
0.7 times speed	0.14 m/s	3	6–9
1 time speed	0.15 m/s	6	6–9

**Table 2:** Summary of experimental results after system improvement.

Theoretical velocity	Actual average speed	Off-track times	FPS
0.5 times speed	0.11 m/s	0	12–15
0.7 times speed	0.14 m/s	0	12–15
1 time speed	0.15 m/s	1	12–15

## Data Availability

No data were used to support this study.
